The article "Place of Angioplasty for Coronary Artery Anomalies With Interarterial Course" was published in 2021. Journal: Front Cardiovasc Med.

# Place of Angioplasty for Coronary Artery Anomalies With Interarterial Course

**DOI:** 10.3389/fcvm.2020.596018

**Published:** 2021-01-18

**Authors:** Pierre Aubry, Xavier Halna du Fretay, Olivier Boudvillain, Philippe Degrell, The ANOCOR Working Group

**Affiliations:** ^1^Bichat Hospital, Department of Cardiology, Paris, France; ^2^entre Hospitalier de Gonesse, Department of Cardiology, Gonesse, France; ^3^Pôle Santé Oréliance, Department of Cardiology, Saran, France; ^4^Centre Hospitalier du Luxembourg, Institut National de Chirurgie Cardiaque et de Cardiologie Interventionnelle, Luxembourg, Luxembourg

**Keywords:** congenital coronary anomaly, anomalous aortic origin, interarterial course, angioplasty, stenting

## Abstract

Few patients with an anomalous aortic origin of a coronary artery (AAOCA) require a correction of this congenital anomaly. Current recommendations offer surgical repair as a first line therapy to prevent a sudden cardiac death as a main objective. However, these guidelines are focused on children and not based on randomized controlled studies. Furthermore, decision-making should be different in an adult population less exposed to the risk of sudden cardiac death. Current practices showed reluctance to offer a surgical treatment for right AAOCA associated with ischemic symptoms or myocardial ischemia. Our aim in this review is to expose the rationale for percutaneous coronary intervention in right AAOCA with interarterial course and to present the published results.

## Introduction

Diagnosis of an anomalous aortic origin of a coronary artery (AAOCA) is not rare in the adult population. A prevalence of 0.8% has been reported with coronary computed tomography angiography (CCTA) (1). Only a part of AAOCA (roughly one-third, i.e., anomalies with an interarterial course between the great vessels) may be associated with cardiovascular events or symptoms (2). The first presentation of these anomalies, so-called AAOCA at risk, is variable, ranging from an incident finding to ischemic symptoms or sudden cardiac death (SCD). The latter is rarely the first event in adults >35 years of age (3). Functional tests are often not able to demonstrate inducible ischemia, even in symptomatic patients (4). When an AAOCA correction is offered, surgical intervention is recommended in current guidelines. But the latter are generally focused on young people (5, 6). The optimal management strategy for older patients with AAOCA at risk remains debated given uncertainties related to the individual risk of SCD or aborted sudden cardiac arrest (SCA), corrected-and not corrected AAOCA natural history, and the risks and failures of the surgery (7). Multidisciplinary teams in charge of AAOCA in the adult population are sometimes faced with a difficult therapeutic choice between a conservative strategy and surgery (8). This review aims to present the possibilities offered by percutaneous coronary intervention (PCI) which may be a realistic alternative to surgery. The PCI management of AAOCA associated with a significant coronary artery disease (CAD) will not be addressed in this review. This work describes the experience and point of view of a French team dedicated to the ANOmalous CORonary arteries: the ANOCOR Working Group.

The article "Place of Angioplasty for Coronary Artery Anomalies With Interarterial Course" was published in 2021. Journal: Front Cardiovasc Med.

## Rationale for Treatment

Several points can be highlighted to understand the rationale for a treatment in the management strategy of AAOCA.

### Sudden Cardiac Death

The relationship between AAOCA and SCD has been established a long time ago (9–12). The risk of SCD leads to anxiety for patients with AAOCA identified at risk, and numerous interrogations for referring practitioners. Post-mortem studies showed that AAOCA is one of the most frequent causes of SCD in athletes (13, 14). Unfortunately, we have no tools to stratify the individual risk of SCD in patients with AAOCA. While the absolute risk is only based on estimations (annual risk of 0.2 and 0.02% for left and right coronary artery, respectively), this risk is particularly low in comparison to the risk of other congenital cardiac diseases identified at-risk of SCD (i.e., hypertrophic cardiomyopathy, arrhythmogenic right ventricular dysplasia, or electric syndromes) (7, 15, 16). The pathophysiological mechanisms that lead to SCD are not fully understood. Physical effort induced-myocardial ischemia is only one of the factors leading to a fatal ventricular arrhythmia. Age <30 years, intense exercise activities, syncope on exertion, left (L)-AAOCA with interarterial course, and maybe myocardial fibrosis scars, are recognized as risk factors for SCD (3, 4, 16, 17). Unfortunately the majority of L-AAOCA at risk is diagnosed postmortem (18). SCD has been described over 35 years of age, but seems particularly rare, especially in patients with right (R)-AAOCA (3). Therefore, the question of primary prevention of SCD should not be asked in the same way for, on the one hand, a young population with L-AAOCA, and on the other hand, older patients with R-AAOCA. After an aborted SCA, a surgical correction is recommended (19), and an internal cardioverter defibrillator is sometimes discussed.

### Ischemic Symptoms and Myocardial Ischemia

A vast majority of AAOCA at risk may remain asymptomatic for a long time, ischemic symptoms, that may mimic a CAD, are possible. AAOCA diagnosis is made by invasive coronary angiography (ICA) or CCTA. Given the difficulty to demonstrate myocardial ischemia by functional non-invasive tests in AAOCA, it seems acceptable to consider non-equivocal symptoms (angina, dyspnea, and syncope, especially on exertion) as ischemic symptoms, even if documented myocardial ischemia is lacking. Symptoms highly suggestive of ischemia are generally included in algorithms for the management of AAOCA (5, 6, 20, 21). Silent myocardial ischemia and severe ventricular arrhythmias must be taken into account in the same way. Considering our knowledge and current guidelines on CAD, medical treatment, PCI, or surgery could be discussed for a symptomatic patient with AAOCA, with the main goals of functional improvement and cardiac events prevention. No controlled randomized study to date has compared the use of anti-ischemic drugs to an alternative strategy in the field of AAOCA. If a SCD may be the first cardiac event, prior ischemic symptoms can be found in nearly half of the cases by questioning the bystanders, entourage or the patient himself in case of aborted SCA (15). Therefore, a correction should always be discussed in AAOCA with ischemic symptoms or documented myocardial ischemia, regardless of age.

The article "Place of Angioplasty for Coronary Artery Anomalies With Interarterial Course" was published in 2021. Journal: Front Cardiovasc Med.

### Current Recommendations

Surgery is recommended as first line therapy in current guidelines for symptomatic AAOCA with interarterial course. In the expert consensus guidelines from the American Association for Thoracic Surgeons (AATS), the authors give a Class 1/Level B indication for any patient with a L-AAOCA at risk, with or without symptoms, or with a symptomatic R-AAOCA at risk (5). In the 2018 AHA/ACC guidelines for the management of adults with congenital heart disease, surgery is recommended (Class 1, Level B-NR) for AAOCA at risk with ischemic symptoms or myocardial ischemia, and is reasonable (Class IIa/Level C-LD) for L-AAOCA at risk without ischemic symptoms or documented myocardial ischemia (6). Surgery or continued observation may be reasonable (Class IIb/Level B-NR) in asymptomatic R-AAOCA without inducible myocardial ischemia or anatomic severity criteria. AATS guidelines don't offer surgery in R-AAOCA without ischemic symptoms or myocardial ischemia. The recent European Guidelines are very close to the Nord American recommendations (21). While the risk of SCD depends strongly on age, the latter is not always taken into account in the current guidelines. To date, none of these recommendations is based on randomized controlled studies. Some authors have pointed out that we don't have objective evidence to strongly recommend surgery in all circumstances. The place of PCI is only addressed in AATS guidelines (5), for adults with high risk for surgery (Class IIb/Level C).

The article "Place of Angioplasty for Coronary Artery Anomalies With Interarterial Course" was published in 2021. Journal: Front Cardiovasc Med.

### Strengths and Weaknesses of Surgery

Several surgical techniques have been developed in the field of AAOCA. Because of the risk of competitive flow, coronary artery bypass grafting is not recommended unless it is associated to a proximal coronary ligation, or in patients with significant CAD beyond the interarterial course. A more anatomic approach is to create a neo-orifice in the appropriate sinus, either by an unroofing procedure with ablation of the intramural aortic segment, or by ostioplasty with patch enlargement (22). A direct reimplantation technique is generally not suitable. Surgical anatomic repair permits to bypass an interarterial course associated or not with an intramural segment. Nevertheless, these therapies carry some risks, and the net benefit against the risk of SCD has not yet been clearly proved. The perioperative mortality is remarkably low at almost zero, with a mild morbidity related to complications of sternotomy and extracorporeal circulation (23, 24). Other complications in relation with surgical technique have been described. Aortic insufficiency by injury of the intercoronary commissure is the main complication observed after an unroofing procedure (25, 26). Early and late complications have also been described with ostioplasty, such as acute occlusion, scarring stenosis, or pseudo-aneurysm (26). The risk of SCD or myocardial ischemia must be heightened against the risk of surgery and the risk of potential late complications. Rarely, aborted SCA has been reported after surgical repair of AAOCA (26).

## Anatomical and Physical Considerations

The nature of coronary narrowings related to atherosclerosis or congenital disease differs greatly.

### Coronary and Aortic Anatomic Considerations

It is admitted that a slit-like orifice is associated with an intramural aortic pathway. However, all AAOCA with interarterial course are not associated with the latter (27, 28). An intramural pathway implies a direct contact between the coronary media and aortic media. Coronary lumen deformation observed in AAOCA with interarterial course should be interpreted as an adaptation of angiogenesis to the limited space between the great vessels, and not as an extrinsic compression. An eccentric deformation with reduction of the lumen area is generally present in AAOAC with an interarterial course (29). Association of an acute connection angle <30° with a ratio >1.5 between long axis and short axis at the narrowest point refers to the presence of an intramural coronary segment embedded within the media of the aorta. The degree of surface reduction varies between 30 and 80%. The length of the interarterial course segment, generally >20 mm, may vary depending of the site of the ectopic orifice. Without intravascular ultrasound (IVUS) guidance, the measurement of the intramural segment length is difficult.

The article "Place of Angioplasty for Coronary Artery Anomalies With Interarterial Course" was published in 2021. Journal: Front Cardiovasc Med.

### Coronary Physical Considerations

Vascular lumen hypoplasia observed on any interarterial segment could be at least partially corrected by stenting. Our experience in CAD related-PCI showed that a lumen oversizing is possible by stenting of coronary arteries whose wall thickness is <0.5 mm. The intramural aortic pathway is associated with specific anatomic features, such as an ellipsoid section and a particularly thick wall (at least 1.0 mm with two media layers) due to the coronary wall embedded into the aortic wall. As a result, the required forces should be greater to optimize the remodeling of an ellipsoid section with an important increase in the minimal diameter and a small decrease in the maximal diameter. A post-PCI circular shape is probably not an achievable target in case of intramural pathways. Due to the non-circular initial shape, mal-apposition of some struts at the edges may be possible. Risks of elastic recoil remain unknown after stenting of a thick arterial wall free of atherosclerosis. Given the proximity of the great vessels, distortion and/or fracture of metallic stents may be a cause of PCI failure with restenosis after several years of dynamic changes. Early in-stent restenosis by intimal hyperplasia remains possible. Aortic wall dissection during catheterization and balloon inflations can be an additional potential risk of the procedure.

### Mechanical Properties of Stents

Uncertainties exist regarding the optimal result of AAOCA stenting. Stents are metallic structures that oppose compressive arterial forces. The mechanical characteristics of stents have not yet been studied in AAOCA. The concept of stenting was developed to improve the results of a balloon dilatation, with a better compression of the atherosclerotic burden and a lesser vascular elastic recoil. Coronary segments with an interarterial course are generally free of atherosclerosis. Basically, the aim of stenting in AAOCA will be performing a vascular remodeling.

## Goals of PCI

There are anatomic and clinical objectives. Structural rigidity of stents may allow them to correct some anatomic features. Ostioplasty of a slit-like orifice and widening of an arterial segment hypoplasia are the expected effects of coronary stenting in this setting. In addition, metallic stents could prevent the presumed interarterial compression and dynamic changes of the intramural lumen morphology during intensive exercise. Clinical objectives are similar to those of the surgery, but in a different manner. The control of ischemic symptoms and the correction of induced myocardial ischemia should be the main objectives of PCI for the target population to be described further. The prevention of major cardiac events such as SCD is of course also expected.

The article "Place of Angioplasty for Coronary Artery Anomalies With Interarterial Course" was published in 2021. Journal: Front Cardiovasc Med.

## PCI Planning

The next part of this review will be focused on the management of R-AAOCA. Indeed, the vast majority of adults for whom a correction is discussed, has R-AAOCA. Moreover, our current knowledge in the field of AAOCA should encourage us to keep surgery as a first line therapy for L-AAOCA, except for adults with high surgical risk.

### Indication of PCI

The evaluation and management of patients with AAOCA at risk should be best discussed by a dedicated multidisciplinary team (cardiologists, radiologists, and surgeons with experience in the AAOCA field). A standardized algorithm, regularly revised, should allow an optimal decision-making for each patient according to the initial presentation and diagnostic work-up. Patients aged over 30 years with R-AAOCA associated with ischemic symptoms and/or documented myocardial ischemia represent the potential population eligible for PCI.

### Non-invasive Imaging Evaluation

Adequate imaging is essential to define anatomic characteristics. Currently CCTA is considered as the best tool to delineate accurately the ostium shape and initial morphology of AAOCA in the adult population (1, 30, 31). A standardized interpretation is recommended including ostial morphology, take-off angle, degree of proximal narrowing compared to the distal part, degree of proximal lumen eccentricity defined as height/width ratio, presence and length of an intramural pathway, and length of the interarterial course. An interarterial course is easy to recognize by CCTA, but the assertion of an intramural pathway can be difficult.

### Techniques of Catheterization

Technical difficulties with catheters are often experienced with R-AAOCA. Given that the initial course is tangential to the aortic wall, canulation and coaxiality, with adequate back-up support, are frequently challenging. A slit-like orifice does not allow a selective canulation. Amplatz left (AL) type catheters are generally the first choice, but Extra-Back-Up (EBU) type catheters can be used. Subselectively advancing of a coronary guide-wire permits enhanced support and higher quality angiographies.

### Invasive Imaging and Physiological Evaluation

Accurate morphological evaluation of AAOCA at risk is crucial. In the 2018 AHA/ACC guideline (6), coronary angiography using catheterization for anatomical and physiological evaluation is recommended in the adult population with AAOCA at risk (Class I, Level C-LD). To date, intravascular ultrasound (IVUS) appears as the imaging technique which provides the best qualitative and quantitative evaluation of the anatomy of AAOCA with an interarterial course (29). IVUS imaging visualizes the aortic wall at the level of an intramural pathway. The ostial shape and coronary narrowing are easily identified by IVUS with a manual pull-back method. Optical Coherence Tomography (OCT) can be used, but an adequate visualization of the orifice shape can be difficult. Physiological evaluation with pressure flow wires could be interesting. However, the Fractional Flow Reserve (FFR) measurement presents some pitfalls in AAOCA. The lack of selective injection needs a hyperemia induced by intravenous adenosine. In addition, the FFR cut-off for AAOCA is unknown. In a series of 25 R-AAOCA (32), a FFR value ≤0.80 was observed in five of the cases (20%). Rest indices such as iFR (instantaneous wave-Free Ratio) remain to be evaluated. So far, we don't have sufficient data to offer a FFR-guided treatment strategy in patients with AAOCA. Nevertheless, a physiological evaluation can be undergone when the decision making is difficult.

The article "Place of Angioplasty for Coronary Artery Anomalies With Interarterial Course" was published in 2021. Journal: Front Cardiovasc Med.

### Techniques of Angioplasty

Remodeling of the lumen appears to be the main objective of PCI. Direct stenting is recommended. However, some operators proposed a pre angioplasty with a cutting-balloon. Empirically, drug-eluting stents with thicker struts and implanted with high pressures (≥20 bars) should be used. The choice of the stent size should be at least the diameter of the coronary segment just downstream of the ectopic course. The stent should be deployed along the entire ectopic course, avoiding too much protrusion into the aorta. PCI guidance by IVUS is recommended for the evaluation of the ectopic segment (diameters, area, and length) and for the control after stenting.

## Results of PCI

### Published Data

The published literature of PCI for AAOCA with an interarterial course remains limited (33–36). Specific treatments of interarterial segment narrowings by PCI should not be confused with percutaneous interventions planned for atherosclerotic stenosis on distal segments of AAOCA with an interarterial course. Several intravascular ultrasound series suggest that the interarterial course of AAOCA is usually free of atherosclerotic disease (32, 37, 38). Doorey et al. reported in 2000 the first experience of PCI for AAOCA with an interarterial course in 12 patients with a mean age of 55 years [44–70] (33). All patients (3 L-AAOCA and 9 R-AAOCA) had abnormal nuclear perfusion imaging tests before stenting. Angiographic success with bare metal stents was obtained in all patients without complications. All patients had normal myocardial functional tests at 6-month follow-up. Angelini et al. have reported in 2015 the largest series with 42 patients with right AAOCA, who underwent PCI because of significant symptoms, positive stress tests, and/or significant stenosis (35). Interestingly, 5 patients had had previous coronary artery bypass grafting to treat R-AAOCA (4 non-functional internal mammary artery grafts and one occluded venous graft). The stenting procedure performed under IVUS guidance was successful in all patients without complications. Drug-eluting stents were used in a majority of cases (39/42). The cross-sectional area increased after stenting from 4.8 to 10.8 mm^2^, reducing the stenosis area from 58 to 8%. Twenty-three (55%) patients underwent follow-up test stressing by nuclear perfusion imaging; only two had perfusion defects in the stented areas. During follow-up (mean 5.0 ± 2.9 years; range 1.1–12.1 years) a significant in-stent restenosis was diagnosed in 4 (10%) patients; two of them had bare metal stents. Three patients underwent in-stent balloon angioplasty and one patient underwent surgery with a mammary artery graft at 6 years for iterative restenosis. Darki et al. reported recently a short series of 4 R-AAOCA treated with drug-eluting stents (36). All patients were symptomatic at presentation. Angiographic success was achieved in all of the cases. All patients were symptom-free after PCI. On the follow-up CCTA (mean duration of 1.4 years), no evidence of stent distortion or fracture was observed. Furthermore, PCI can be used to treat some surgery failures, such as acute occlusion or scarring stenosis (26).

The article "Place of Angioplasty for Coronary Artery Anomalies With Interarterial Course" was published in 2021. Journal: Front Cardiovasc Med.

### ANOCOR Working Group Experience

Based on this experience reported in the literature, the ANOCOR Working Group has started since 2014 a prospective registry (ANOCOR Stenting) of patients with R-AAOCA and treated by PCI with stenting (39). All patients were discussed in monthly multidisciplinary meetings. A decision-making algorithm (Figure 1) was applied for the evaluation and management of patients with AAOCA. Aborted SCA was considered an exclusion criteria. A percutaneous treatment by stenting was proposed for patients with R-AAOCA referred to the expert group according to predefined criteria: age >30 years (except for patients with a left coronary dominance), ischemic symptoms or documented myocardial ischemia, interarterial course). All patients underwent invasive CA and CCTA. Additional evaluation by IVUS or OCT was recommended. Clinical follow-up was scheduled at 6, 12, and 60 months by phone contact. Systematic CCTA and functional testing with imaging were proposed between 6 and 12 months. Patients continued dual antiplatelet therapy for at least 6 months. Seventeen patients (mean age 51 years) were prospectively included between 2014 and 2019. Two patients had acute coronary syndrome, twelve had stable angina, two were asymptomatic with a positive stress test and one had syncope. An intramural segment was identified in more than half of the patients. Stenting was successful with residual angiographic stenosis <30% in all of the procedures, 47% radial access, 94% of drug-eluting stents, mean stent diameter 3.5 mm, mean stent length 25 mm, mean fluoroscopic time of 19 min, and >80% of IVUS or OCT guidance. Coronary morphology is modified by stenting with a trend toward a more circular lumen (Figure 2). However, the latter remains generally ovoid after stenting of an intramural pathway. There were no periprocedural complications. Clinical follow-up at 6 months was uneventful in all but one patient requiring a new hospitalization at 5 months for persistent angina reported to be a vasospastic angina. Two patients had in-stent restenosis between 6 and 12 months post-procedure needing a new PCI. No stent distortion was observed on follow-up CCTA (Figure 2).

The article "Place of Angioplasty for Coronary Artery Anomalies With Interarterial Course" was published in 2021. Journal: Front Cardiovasc Med.

**Figure 1:** Algorithm to evaluate and manage patients with anomalous aortic origin of a coronary artery (AAOCA). ^1^Optional.

**Figure 2:** **(A)** Example of angioplasty with stenting of a right AAOCA (pre-PCI, stent deployment, post-PCI); **(B)** angioplasty with stenting under IVUS guidance of a right AAOCA associated with an intramural pathway (pre-PCI, stent deployment, post-PCI); **(C)** CCTA images of a right AAOCA treated by angioplasty with stenting (pre-PCI and post-PCI at-6 month). AAOCA, anomalous aortic origin of a coronary artery; CCTA, coronary computed tomography angiography; PCI, percutaneous coronary intervention; IVUS, intravascular ultrasound.

## Limitations and Strengths of PCI

As the surgery, we don't know the long-term outcomes of the management of AAOCA with PCI (Table 1). The strengths of the latter in comparison with the surgery are those usually observed in the CAD treatment, with a shorter hospital stay and less post procedural adverse events with the percutaneous approach. In addition, the latter may be accomplished by the vast majority of interventional cardiologists. In opposite, few cardiac surgeons are able to repair AAOCA.

**Table 1:** Main characteristics of patients included in series of AAOCA treated by angioplasty with stenting.

**References**	**AAOCA type and number**	**Mean age years**	**BMS/DES number**	**Angiographic success (%)**	**Mean follow-up years**	**In-stent restenosis number (%)**	**Stent compression number (%)**	**Sudden cardiac death number**
Doorey et al. (33)	3 Left/9 Right	56	12/0	100	0.5	3 (25)	1 (8)	0
Angelini et al. (35)	42 Right	48	3/39	100	5.0	4 (10)	0	0
Degrell et al. (39)	17 Right	51	1/16	100	2.0	2 (12)	0	0
Darki et al. (36)	4 Right	64	0/4	100	8.5	NA	0	0

*AAOCA, anomalous aortic origin of a coronary artery; BMS, bare metal stent; DES, drug eluting stent*.

The article "Place of Angioplasty for Coronary Artery Anomalies With Interarterial Course" was published in 2021. Journal: Front Cardiovasc Med.

## Discussion

R-AAOCA constitutes a major part of congenital coronary anomalies possibly responsible for ischemic symptoms or myocardial ischemia. The management of patients with R-AAOCA remains controversial in the adult population. Current guidelines recommend a surgical repair for R-AAOCA with evidence of ischemia. A very low risk of SCD, the lack of randomized controlled studies and scarcity of long-term data may explain the low rate of surgically treated patients. A percutaneous approach may provide an interesting alternative in a selected adult population. Our experience and that of others showed that stenting of an interarterial course was feasible and safe without risks of aortic or coronary dissection. Arterial remodeling associated with a significant increase in lumen area can explain symptom relief and myocardial ischemia resolution. The design of the abovementioned studies did not allow the evaluation of the impact of stenting on SCD risks. We should consider the risk of in-stent restenosis (about 10% of cases) that can be difficult to treat in case of strut protruding into the aorta. An extrinsic compression of a metallic stent placed between the great vessels has not been reported yet. More information is needed with longitudinal studies of a larger population, longer clinical and CCTA follow-ups, and prospective data collection. In the future, a percutaneous option for the treatment of selected R-AAOCA should be considered in the decision-making algorithm in specialized centers.

## Author Contributions

PA wrote the initial draft of the review and supervised corrections. PD contributed substantially to the content of the review. XHF and OB reviewed all drafts, providing revisions. All authors agree to be accountable for the content of the work.

## ANOCOR Working Group

Dr. Pierre Aubry, Dr. Paul Barragan, Dr. Olivier Boudvillain, Dr. Philippe Commeau, Dr. Philippe Degrell, Dr. Patrick Dupouy, Reza Farnoud, Dr. Xavier Halna du Fretay, Dr, Fabien Hyafil, Dr. Jean-Michel Juliard, Prof. Jean-Pierre Laissy, Dr. Damien Millischer, Prof. Pascal Motreff, Dr. Mohammed Nejjari, Prof. Phalla Ou.

## Conflict of Interest

The authors declare that the research was conducted in the absence of any commercial or financial relationships that could be construed as a potential conflict of interest.

## Abbreviations

AAOCA: anomalous aortic origin of a coronary artery
AATS: American Association for Thoracic Surgeons
ANOCOR: ANOmalous CORonary arteries
CAD: coronary artery disease
CCTA: coronary computed tomography angiography
ICA: invasive coronary artery
IVUS: intravascular ultrasound
FFR: fractional flow reserve
PCI: percutaneous coronary intervention
SCA: sudden cardiac arrest
SCD: sudden cardiac death.
